RETRACTED

# Frequency and Predictors of Acute Kidney Injury in Patients With Acute Coronary Syndrome in a Tertiary Care Hospital: A Retrospective Study

**DOI:** 10.7759/cureus.21869

**Published:** 2022-02-03

**Authors:** Hemanth Kumar, Daniyal Jilanee, Shivani M Mehta, Amna Gul, Syed Muhammad Huzaifa Shah, Sumaira Saleem, Maria Binte Sarfraz, Syed U Ashraf, Sher Wali

**Affiliations:** 1 Medical School, Maharajah's Institute of Medical Science, Nellimarla, IND; 2 Medical School, Liaquat National Hospital and Medical College, Karachi, PAK; 3 Medical School, Xavier University School of Medicine, Oranjestad, ABW; 4 Medical School, Ziauddin University, Karachi, PAK; 5 Medical School, Dow Medical College, Dow University of Health Sciences, Karachi, PAK; 6 Department of Physiology, Army Medical College, National University of Medical Sciences, Rawalpindi, PAK; 7 Internal Medicine, Dow International Medical College, Dow University of Health Sciences, Karachi, PAK; 8 Research, Indus Hospital & Health Network, Karachi, PAK

**Keywords:** renal dysfunction, predictors, frequency, acute coronary syndrome, acute kidney injury

## Abstract

Introduction

Acute kidney injury (AKI) is a complex condition marked by rapid deterioration of renal function (within hours or days), with clinical symptoms ranging from a minor rise in serum creatinine to anuric renal failure needing renal replacement therapy. AKI is one of the complications of acute coronary syndrome (ACS). This study aims to determine the frequency of AKI among patients with ACS and identify its predictors.

Method

This study is a retrospective observational study conducted at the Dow University of Health Sciences, a tertiary care hospital located in Karachi, Pakistan. This study was conducted from January 2020 to June 2021. All patients aged 18-75 years admitted with ACS and admitted for more than 48 hours were included in the study. A pre-set questionnaire was used to collect data from the hospital management information system (HMIS).

Results

The frequency of AKI among patients with ACS was 24.18%. The factors associated with AKI among patients with ACS on multivariable logistic regression included the age of patients (odds ratio (OR) = 1.04, p-value = 0.018), having diabetes mellitus (OR = 2.33, p-value = 0.031), admission Killip ≥ II (OR = 2.12, p-value = 0.041), previous history of myocardial infarction (MI) (OR = 3.64, p-value = 0.001), baseline glomerular filtration rate (GFR) (OR = 0.94, p-value = 0.001), in-hospital ejection fraction (EF) (OR = 0.93, p-value = 0.001), and serum creatinine at admission (OR = 1.02, p-value = 0.001).

Conclusion

Age, comorbidities including diabetes mellitus and previous history of MI, admission Killip ≥ II, baseline GFR, in-hospital EF, and serum creatinine level at admission are significant independent predictors of AKI in patients with ACS.

RETRACTED

## Introduction

Acute kidney injury (AKI) is a complex condition marked by rapid deterioration of renal function (within hours or days), with clinical symptoms ranging from a minor rise in serum creatinine to anuric renal failure needing renal replacement therapy [1]. Its most severe manifestation is cardiorenal syndrome (CRS) type 1, which is defined as "an acute worsening of heart function leading to AKI or kidney dysfunction." It is a complication of acute heart failure (AHF) or acute coronary syndrome (ACS). It is associated with an increased duration of hospital stay and mortality [2]. Several studies have shown that acute renal dysfunction occurs in one of five cases of ACS, and it is one of the leading predictors of cardiovascular complications [3,4].

In patients with ST-elevation myocardial infarction (STEMI) and non-ST-elevation myocardial infarction (NSTEMI), systemic hypoperfusion causes renal ischemia due to acute left ventricular (LV) systolic failure, which appears to be a key pathophysiological mechanism causing AKI. Other important factors that contribute to AKI included neurohumoral activation, increased sympathetic activity, hyperglycemia, nephrotoxic drugs, and hypovolemia [5,6]. The risk factors responsible for AKI development include anemia, dehydration, diabetes mellitus, older age, and baseline chronic kidney disease [7,8].

It is quite surprising that recent guidelines and several cardiology textbooks have not drawn much attention to AKI in patients with ACS [9]. However, recommendations are there to manage potential but relatively rare complications of ACS, such as Dressler pericarditis or papillary muscle rupture. Not much information is given about AKI, despite the fact that its incidence is high as 30% [10].

Most patients with AKI are not followed after discharge from the hospital. Thus, it is important to conduct research for early identification of patients at high risk for acute renal impairment that is important to improve outcomes in patients with ACS. No study was conducted in Pakistan that determines the incidence of AKI among patients with ACS as the characteristics of the Pakistani population are different from people in developed countries. Thus, this study aims to determine the frequency of AKI among patients with ACS and identify its predictors.

## Materials and methods

Methodology

This study is a retrospective observational study conducted at the Dow University of Health Sciences, a tertiary care hospital located in Karachi, Pakistan. This study was conducted from January 2020 to June 2021. All patients with the age of 18-75 years admitted with ACS and admitted for more than 48 hours were included in the study.

RETRACTED

Eligibility criteria

Patients with all kinds of ACS, including ST-elevation myocardial infarction (STEMI) and non-ST elevation myocardial infarction (NSTEMI), were included in the study. Patients were excluded if they had known neoplastic, hepatic, autoimmune, or infectious diseases. Patients with a kidney transplant, existing diagnosis of chronic kidney disease, and previous or current dialysis were also excluded from the study. Patients with missing data were also not included in the final analysis.

Data collection

A pre-set questionnaire was used to collect data from the hospital management information system (HMIS). Demographic and clinical data, including age, gender, smoking status, comorbidities, and body mass index (BMI), were obtained. BMI was calculated by dividing weight (kg) and the square of height (m).

Outcome variable and independent variables

According to the Kidney Disease: Improving Global Outcomes (KDIGO) guidelines, AKI was defined as an increase in serum creatinine by 0.3 mg/dL or more within 48 hours or an increase in serum creatinine to 1.5 times the baseline or more within the last seven days or urine output of less than 0.5 mL/kg/hour for six hours [11]. We did not have urine output data of patients, so AKI was just defined in the current study on the basis of an increase in serum creatinine. The baseline creatinine was defined as the lowest creatinine during hospitalization that could not be explained by fluid resuscitation, overload, or dialysis. It was sustained for more than 72 hours or until the patient was discharged [11].

Data related to laboratory values, including hemoglobin, total cholesterol, triglycerides, serum creatinine, and in-hospital ejection fraction (EF), were obtained from the HMIS. The serum creatinine at hospital admission and the daily serum creatinine during the patient stay at the coronary care unit were measured for all patients as part of patients' daily routine care. The estimated glomerular filtration rate (GFR) was estimated using the Cockcroft-Gault formula to determine the filtration function of the kidneys [12]. Heart failure severity was assessed using Killip classification. Patients were categorized as Killip class II if they had pulmonary congestion, class III if they had pulmonary edema, or class IV if they had cardiogenic shock [13].

Statistical analysis

Analysis was done using STATA version 16.0. Mean and standard deviation were presented for continuous variables, while frequency and percentage were calculated for categorical variables. Categorical data were compared between patients with AKI and patients without AKI using the chi-square test and independent t-test for categorical and continuous variables, respectively. The identification of the independent predictors of AKI was done using multivariable logistic regression analysis with stepwise selection of variables. The results of the analysis were presented as odds ratio (ORs) and 95% confidence intervals (CIs). A p-value of less than 0.05 was considered significant.

RETRACTED

## Results

Overall, 360 patients were admitted to the coronary care unit of Dow University of Health Sciences. Ninety patients (25%) did not fulfill the eligibility criteria, while the data of 26 patients (7.22%) were incomplete. The data of 244 patients (67.78%) were included in the final analysis. The baseline characteristics of 244 patients with STEMI and patients with NSTEMI admitted to the coronary care unit are shown in Table 1. Out of 244 patients enrolled in the study, 59 (24.18%) developed AKI. Significant differences were obtained between the AKI and non-AKI groups. The mean age in the AKI group (68.08 + 10.86) is significantly higher than the mean age in the non-AKI group (63.12 + 11.17) (p-value = 0.003). Significant differences were obtained between the non-AKI and AKI group in diabetes mellitus (21.08% versus 47.46%, p-value = 0.001) and previous history of MI (p-value = 0.001) and admission Killip score ≥ II (p-value = 0.001).

**Table 1:** General clinical characteristics of patients depending on the presence of acute kidney injury * Significant at p-value < 0.05 ^ Mean (standard deviation) BMI: body mass index; MI: myocardial infarction

Variables	Categories	Non-AKI (n (%))	AKI (n (%))	P-value
Age in years^		63.12 (11.17)	68.08 (10.86)	0.003*
Gender	Male	131 (70.81)	48 (81.36)	0.111
	Female	54 (29.19)	11 (18.64)	
BMI	Normal	46 (24.86)	20 (33.90)	0.164
	Overweight	83 (44.86)	28 (47.46)	
	Obese	56 (30.27)	11 (18.64)	
Diabetes mellitus	No	146 (78.92)	31 (52.54)	0.001*
	Yes	39 (21.08)	28 (47.46)	
Preexisting hypertension	No	5 (2.70)	1 (1.69)	0.202
	Yes	180 (97.30)	58 (98.31)	
Currently smoking	No	118 (63.78)	45 (76.27)	0.076
	Yes	67 (36.22)	14 (23.73)	
Diagnosis	STEMI	111 (60)	38 (64.41)	0.546
	NSTEMI	74 (40)	21 (35.59)	
Previous history of MI	No	140 (75.68)	30 (50.85)	0.001*
	Yes	45 (24.32)	29 (49.15)	
Admission Killip ≥ II	No	107 (57.84)	23 (38.98)	0.001*
	Yes	78 (42.16)	36 (61.02)	

Table 2 shows the laboratory results on admission and hospital stay of 244 patients enrolled in this study. Serum creatinine at admission and triglycerides were significantly higher in the AKI group compared with the non-AKI group (p-value < 0.05). On the other hand, hemoglobin, baseline GFR, and in-hospital EF were significantly higher in the non-AKI group than in the AKI group (p-value < 0.05).

RETRACTED

**Table 2:** Laboratory values of patients depending on the presence of acute kidney injury Presented as mean (standard deviation) * Significant at p-value < 0.05 GFR: glomerular filtration rate; EF: ejection fraction

Variable	Non-AKI	AKI	P-value
Hemoglobin (g/L)	142.76 (20.41)	130.01 (26.45)	0.001*
Total cholesterol (mmol/L)	4.85 (1.36)	4.55 (1.46)	0.147
Triglycerides (mmol/L)	1.52 (0.75)	1.78 (0.84)	0.034*
Admission serum creatinine (µmol/L)	101.60 (31.05)	190.05 (154.94)	0.001*
In-hospital EF (%)	51.19 (6.98)	47.22 (8.34)	0.001*
Baseline GFR (mL/minute/1.73 m^2^)	62.80 (22.17)	39.63 (21.92)	0.001*

All variables significant in univariate analysis were included in multivariable logistic regression analysis using a stepwise approach, and the results are presented in Table 3. The variables significantly associated with AKI among patients with ACS included the age of patients (OR = 1.04, p-value = 0.018), having diabetes mellitus (OR = 2.33, p-value = 0.031), admission Killip ≥ II (OR = 2.12, p-value = 0.041), previous history of MI (OR = 3.64, p-value = 0.001), baseline GFR (OR = 0.94, p-value = 0.001), in-hospital LVEF (OR = 0.93, p-value = 0.001), and serum creatinine at admission (OR = 1.02, p-value = 0.001).

**Table 3:** Significant factors associated with AKI among patients with ACS (multivariable logistic regression analysis) OR: odds ratio; CI: confidence interval

Variable	Categories	OR (95% CI)	P-value
Age		1.04 (1.01–1.07)	0.018
Diabetes mellitus	No		
	Yes	2.33 (1.07–5.03)	0.031
Admission Killip ≥ II	No		
	Yes	2.12 (1.03–4.32)	0.041
Previous history of MI	No		
	Yes	3.64 (1.74–7.62)	0.001
Baseline GFR		0.94 (0.93–0.97)	0.001
In-hospital EF		0.93 (0.89–0.97)	0.001
Admission serum creatinine		1.02 (1.01–1.05)	0.001

## Discussion

Acute renal dysfunction is one of the common complications that can develop in patients with ACS [14]. In our study, acute kidney injury developed in 24.18% of the patients. As per the study conducted by Zhunuspekova et al., 23.2% of patients developed acute kidney dysfunction [15].

In our study, AKI was significantly associated with AHF on admission that was assessed using the Killip classification and decreased LVEF. Decreased EF indicated the loss of contractility because of myocardial necrosis and acute ischemia [16]. A study conducted by Sinkovič et al. also found that decreased EF was associated with Killip class ≥ II, particularly in patients who developed AKI [17]. Different clinical prospective studies have shown that increased NT-proBNP, associated with a cardiorenal syndrome, venous congestion, hyponatremia, and hypotension, is one of the risk factors for AKI [18,19]. AHF causes a decrease in renal blood flow that activates the renin-angiotensin-aldosterone systems and induces ventricular remodeling [20].

RETRACTED

Our study has found that the frequent comorbidities in patients with AKI were the previous history of MI and diabetes mellitus. It suggests that both of these comorbidities can contribute to AKI in patients with ACS. Similar findings were obtained by the study conducted by Sinkovič et al. [17]. A study conducted by Shiyovich et al. found that patients with diabetes mellitus have a higher risk of developing AKI when admitted with ACS [21]. Diabetes mellitus is associated with increased oxidative stress and reactive oxygen species (ROS) arbitrated by enhanced activity of reduced nicotinamide adenine dinucleotide phosphate (NADPH) oxidase and increased mitochondrial superoxide [22]. Moreover, diabetes mellitus is associated with enhanced consumption of renal oxygen via the enhancement of a load of several ion pumps [23].

Several studies have shown that chronic kidney disease or renal failure is an independent predictor of AKI in patients with ACS [24]. In our study, the baseline serum creatinine level was the risk factor for AKI. A study conducted by Zhunuspekova et al. also found baseline serum creatinine level as the leading risk factor of AKI in patients with ACS [15]. Age, creatinine, and left ventricular ejection fraction are all parameters in the ACEF risk model (2009), which is used to assess the risk of unfavorable cardiovascular events in patients after surgical and percutaneous myocardial revascularization. The study conducted by Ranucci et al. found that there was an increase in the frequency of the composite endpoint, which included mortality from heart disease, acute myocardial infarction, or stroke, at creatinine levels above 2 mg/dL (177 mol/L) [25].

AKI is one of the serious complications of ACS that can cause serious complications such as malignant arrhythmias and cardiogenic shock [8]. Considering the current study's findings and taking into account that no well-developed medical therapies are available, secondary preventive measures need to be implemented that aim to improve outcomes among survivors of AKI [26]. Besides this, nephrologists should follow these patients, and cardiologists should do an early assessment of all patients, especially patients at high risk of developing AKI, including patients with diabetes and patients with a history of MI, to prevent AKI and other serious complications from occurring.

The current study has certain limitations. Firstly, this study was conducted using a retrospective design, and it was a single-center study. Secondly, due to increased serum creatinine levels not being measured in patients who died during the first few hours of hospital admission, the incidence of AKI may have been underestimated. Thirdly, we did not classify patients as per the severity of AKI. In addition, we do not have data regarding whether patients recovered or not.

RETRACTED

## Conclusions

Our study has found that age, comorbidities including diabetes mellitus and previous history of MI, admission Killip ≥ II, baseline GFR, in-hospital LVEF, and serum creatinine level at admission are significant independent predictors of AKI in patients with ACS. To prevent AKI in patients with ACS, secondary preventive measures need to be implemented. Proper follow-up of patients with AKI needs to be done to prevent any complications in these patients. High-risk patients need to be identified at an early stage, and guidelines need to be developed regarding the prevention and management of AKI among patients with ACS.
